RETRACTED

# Effect of Acupuncture and Rehabilitation Therapy on the Recovery of Neurological Function and Prognosis of Stroke Patients

**DOI:** 10.1155/2022/4581248

**Published:** 2022-02-22

**Authors:** Lanping Fu, Fei Wang, Zhiyi Ma, Jin Zhang, Wuzhong Xiong, Le Wang

**Affiliations:** ^1^Department of Acupuncture and Moxibustion, Wuhan Hospital of Traditional Chinese Medicine, Wuhan, 430000 Hubei Province, China; ^2^Stroke Department of Wuhan Hospital of Traditional Chinese Medicine, Wuhan, 430000 Hubei Province, China; ^3^Department of Rheumatology, Wuhan Hospital of Traditional Chinese Medicine, Wuhan, 430000 Hubei Province, China; ^4^Department of Orthopedics, Wuhan Hospital of Traditional Chinese Medicine, Wuhan, 430000 Hubei Province, China; ^5^Department of Internal Medicine, Wuhan Hospital of Traditional Chinese Medicine, Wuhan, 430000 Hubei Province, China

## Abstract

**Background:**

Stroke is a common cerebrovascular disease among the middle-aged and elderly, which can lead to a series of neurological disorders. Acupuncture is an important part of traditional Chinese medicine, with great value in improving the neurological deficits of stroke patients. In addition, rehabilitation therapy is also of great significance for alleviating the neurological deficits of patients and improving their activities of daily living.

**Objective:**

To explore the effect of acupuncture and moxibustion combined with rehabilitation therapy on the recovery of neurological function and prognosis of stroke patients.

**Methods:**

The case data of 100 stroke patients treated in the Wuhan Hospital of Traditional Chinese Medicine from January 2019 to July 2021 were analyzed retrospectively. According to the treatment plan patients received, they were divided into the following two groups: an observation group (*n* = 52) treated with acupuncture combined with rehabilitation therapy and a control group (*n* = 48) treated with rehabilitation therapy alone. The two groups were compared in terms of the following items: therapeutic efficacy, plasma levels of cortisol (Cor) and neuropeptide Y (NPY), nerve function, motor function, balance ability, self-care ability, swallowing function, negative emotions, and quality of life.

**Results:**

The therapeutic effect of the observation group was significantly higher than that of the control group (*P* < 0.05). The levels of Cor and NPY, as well as the neurological function, motor function, balance ability, self-care ability, swallowing function, and negative emotions, were not significantly different between the two groups before treatment (*P* > 0.05). While after intervention, all the above indexes improved in both groups, with better improvements in the observation group compared with the control group (*P* < 0.05). And the various dimensions concerning the quality of life of patients were also significantly better in the observation group when compared with the control group.

RETRACTED

**Conclusion:**

Acupuncture of traditional Chinese medicine combined with rehabilitation therapy has outstanding effects in stroke treatment and can effectively improve the neurological function, prognosis, and quality of life of patients, which is worthy of clinical promotion.

## 1. Introduction

Stroke, a cerebrovascular disease that occurs frequently in middle-aged and elderly people, is a sudden attack of disturbance of cerebral blood circulation, with the characteristics of fast onset, rapid development, and many complications [1, 2]. Relevant studies have shown that the incidence of neurorelated dysfunction, including language disorders, limb sensation, and movement disorders, accounts for about 75% of all stroke patients [3, 4]. The mortality and disability rate of stroke are high in clinical practice, which seriously affects patients' quality of life and their health both physically and psychologically. Therefore, early and effective targeted treatment for stroke patients after onset is of great significance to the prevention of complications and the improvement of patient prognosis [5, 6].

Western medicine, the main clinical treatment for stroke, can improve clinical symptoms and inhibit disease progression to a certain extent. However, due to the high disability rate of patients with neurological impairment, the overall effect of western medicine treatment in long-term clinical practice is not ideal, and the prognosis of patients is poor, which seriously affects the life quality of patients [7]. As an important part of rehabilitation medicine, rehabilitation therapy, on the other hand, can improve the coordination ability, balance ability, and movement control ability of patients through a series of rehabilitation exercise activities, which is of great significance to alleviate patients' neurological deficits and improve their self-care ability [8]. In addition, traditional Chinese medicine believes that stroke is caused by various factors such as irregular menstruation, disorder of qi and blood, and blockage of meridians [9]. Acupuncture is an essential and irreplaceable part of traditional Chinese medicine, which applies needles to stimulate the corresponding acupoints of the patient's body based on the relevant laws of meridian points, veins, and viscera on the body surface, so as to dredge the meridians and collaterals and relieve the symptoms. It also has the advantages of simple implementation and low complication rate, which is of great value in alleviating the neurological deficit of stroke patients [10, 11]. The National Institutes of Health Stroke Scale (NIHSS) [12], which is the most extensively used clinical scale to evaluate patients with acute stroke, was used as the primary outcome measure in this study. The scale has the advantages of simplicity and high efficiency, through which clinicians can also accurately evaluate patients.

RETRACTED

Given that there are currently few studies on the effects of acupuncture combined with rehabilitation therapy on the neurological function of stroke patients, this study conducted a detailed discussion on it, aiming to provide more references for the treatment of stroke patients.

## 2. Materials and Methods

### 2.1. Clinical Information

The case data of 100 stroke patients who came to the Wuhan Hospital of Traditional Chinese Medicine from January 2019 to July 2021 were analyzed retrospectively. According to different treatment plans, 52 patients treated by acupuncture combined with rehabilitation therapy were included in the observation group, and 48 patients who received rehabilitation therapy alone were included in the control group. Inclusion criteria were as follows: patients who were diagnosed with stroke by MRI or cranial CT and met the diagnostic criteria for stroke [12], patients who had an attack within 7 days with stable vital signs, patients aged 55-75 years, and patients who agreed to participate in the study. Exclusion criteria were as follows: (1) patients with consciousness disorders, (2) patients with severe trauma, (3) patients with malignant tumors, (4) patients with organic damage to vital organs other than the brain, such as liver and kidney, and (5) patients who might faint during acupuncture. All patients agreed to participate in the study with a written informed consent signed. This experiment was approved by the Ethics Committee of Wuhan Hospital of Traditional Chinese Medicine and conformed to the Declaration of Helsinki.

### 2.2. Therapeutic Plans

Both groups received conventional treatments, which mainly included protecting brain cells, improving brain microcirculation, relieving cerebral edema, lowering blood pressure, and preventing infection and symptomatic treatment such as lowering intracranial pressure for those with excessive intracranial pressure. Limb function training was started 48 hours after the patient had clear consciousness, stable vital signs, and no progression or deterioration of neurological-related symptoms. The training started with the simplest movements and progressed to more complex ones, the amount of exercise increased gradually, and the training mode shifted from passive to active. Repetitive exercises were performed on the affected side with lying position and supine position, respectively. Functional training of the affected side limbs was enhanced to increase muscle tension, then repeated exercises were continued, and the range of activities was gradually expanded according to the situation. Specific training was as follows: (1) placement of nonaffected limbs: patients were asked to place the limbs in a normal functional position, with the affected side's shoulder joint rotated outwardly, the elbow joint kept in a stretched position, the hip joint properly adducted, the ankle joint in the dorsal flexion position, and the knee joint properly flexed. (2) Joint function training: patients were instructed to drive the affected joint with the uninhibited limb and perform active joint exercises and passive joint exercises appropriately. (3) Posture transfer: patients were asked to lie down, then sit, and then maintain a standing position, following the principle of systematization. (4) Balance training: patients were instructed to perform training such as trunk scoliosis and rotation and then gradually guided to carry out walking and stair climbing training. (5) Swallowing function training: patients were instructed to perform mouth-opening, mouth-closing, tongue-out, puffing, and swallowing exercises in order to improve their swallowing function. Limb function training was performed once a day for 30 minutes for 1 month.

RETRACTED

Patients in the observation group were treated with acupuncture and moxibustion on the basis of the above treatment. According to the principle of treatment and acupuncture based on syndrome differentiation, the acupuncture points such as Jianyu, Hegu, Huantiao, Shousanli, Yanglingquan, Zusanli, Taichong, Shenshu, Dazhui, Twelve Jing, Weizhong, and Waiguan were selected for patients with hemiplegia; for those with speech dysfunction, acupoints such as Yamen, Lianquan, and Tongli were selected; for patients with crooked mouth, acupuncture points such as Cheekche, Taichong, Renzhong, Hegu, and Dilun were selected. The specific methods of acupuncture and moxibustion were as follows: routine disinfection of the skin at the puncture site was performed on patients in the sitting-supine position. It was worth noting that the Neiguan acupoint adopted the reduction method, Sanyinjiao acupoint adopted the replenishing method, Shuigou acupoint adopted the cough method, and Weizhong and Chize acupoints adopted the straight needling method. The lifting-thrusting method was adopted to make patients feel twitching and swelling on the limbs. The rest of the acupoints was operated according to the method of invigorating and reducing deficiency, and bilateral acupoints were selected for treatment, focusing on the acupoints on the affected side, with a depth of 0.5 to 1.0 cun. After acupuncture, the needle was left for 25 to 30 minutes. The treatment was performed once a day with a total of 4 courses of treatment (7 days as a course of treatment).

RETRACTED

### 2.3. Outcome Measures

(1) We evaluated and compared the therapeutic effects of two groups of patients and divided them into markedly effective: the patient's neurological deficit score was ≥81% after treatment; effective: the patient's neurological deficit score was between 36% and 80% after treatment; ineffective: the neurological deficit score of the patient was ≤35% after treatment. (2) The National Institutes of Health Stroke Scale (NIHSS) [13] was used to evaluate the neurological impairment of patients before and after treatment. The higher the score, the more severe the neurological impairment. (3) We compared the plasma levels of cortisol (Cor) (Shanghai Chaoyan Biotechnology Co., Ltd.) and neuropeptide Y (NPY) (Shanghai Xinyu Biotechnology Co., Ltd.) of patients in two groups before and after treatment. Before and after treatment, 5 ml of fasting venous blood was collected from patients into vacuum blood collection tubes, and the plasma was collected after anticoagulation treatment. Radioimmunoassay was used to detect plasma levels of Cor and NPY. (4) The simplified Fugl-Meyer Assessment (FMA) scale [14] was used to evaluate the motor function of the limbs, with a total score of 100 points. Higher scores suggest better motor function of the limbs. (5) The Barthel index [15] was utilized to assess patients' activities of daily living before and after treatment from the areas of feeding, bathing, dressing, grooming, urinating ability, defecation ability, toilet use, transfers (bed to chair and back), walking, and stairs, with a total of 10 items and a full score of 100 points. Higher scores indicate better activities of daily living. (6) The Berg Balance Scale (BBS) [16] was used to assess the balance ability of patients, including 14 items and each of which uses a five-level score (0 to 4 points) with a total score of 56 points. Higher scores indicate better balance. (7) The M.D. Anderson Dysphagia Inventory (MDADI) [17] was to evaluate the swallowing function of patients before and after treatment. The scale was divided into four dimensions: global, emotional, functional, and physical. Likert's 5-level score was adopted for measuring: 1 point: very agree and 5 points: very disagree. The global dimension was scored separately, and the scores of other dimensions were added together. The average value was multiplied by 20 to get the total score of the scale. The score range is 0-100 points. The higher the score, the better the swallowing function. (8) The Self-Rating Depression Scale (SDS) and Self-Rating Anxiety Scale (SAS) [18] were to evaluate and compare the negative emotions of patients before and after treatment. (10) The World Health Organization Quality Of Life- (WHOQOL-) 100 Scale [19] was to evaluate the life quality of patients after treatment from five dimensions: physiology, psychology, social relationships, living conditions, and level of independence. Higher scores suggest better quality of life.

RETRACTED

### 2.4. Statistical Methods

SPSS 19.0 statistical software (IBM) was used for statistical analysis of the data, and GraphPad 7 was used for image rendering. Count data were recorded in the form of number of cases and percentages (%), and the chi-square test was used for analysis. For measurement data, paired *t*-test was used for comparisons before and after treatment and independent samples *t*-test for intergroup comparisons. *P* < 0.05 indicated that the difference was of statistical significance.

## 3. Results

### 3.1. Comparison of General Information

There were no significant differences in general information such as gender, age, and body mass index (BMI) between the two groups (*P* > 0.05), suggesting comparability (Table 1).

### 3.2. Comparison of Therapeutic Effect between Groups

The number of patients in the observation group who were markedly effective, effective, and ineffective after treatment was 30, 20, and 2, respectively, with an overall response rate (ORR) of 96.15%. while the number of patients in the control group was 22, 16, and 10, respectively, with an ORR of 79.17%. The results showed that the observation group had a higher effective rate than the control group (*P* < 0.05) (Table 2).

### 3.3. Comparison of Neurological Deficit Scores before and after Treatment between Groups

No significant difference was observed in the NIHSS scores between the two groups before treatment (*P* > 0.05); while after treatment, the NIHSS score of both groups was reduced, and the score in the observation group (11.24 ± 1.12) was lower than that in the control group (17.19 ± 1.23) (*P* < 0.05) (Table 3).

### 3.4. Comparison of Plasma Cor and NPY Levels before and after Treatment between Groups

The plasma levels of Cor and NPY decreased in both groups after treatment and were lower in the observation group compared with the control group (*P* < 0.05) (Figure 1).

### 3.5. Comparison of Fugl-Meyer Assessment (FMA) for Motor Function and Barthel Index for Activities of Daily Living before and after Treatment between Two Groups

Before treatment, the FAM and Barthel scores of the observation group were not significantly different from those of the control group (*P* > 0.05). While after treatment, the FAM score (46.28 ± 4.06) and Barthel score (85.67 ± 4.96) increased significantly in the observation group compared with the control group (*P* < 0.05) (Figure 2).

RETRACTED

### 3.6. Comparison of BBS Scores before and after Treatment between Two Groups

No significant difference was observed in the BBS score between the two groups before treatment (*P* > 0.05). While the BBS score increased significantly in both groups after treatment, the score in the observation group was higher than that in the control group (*P* < 0.05) (Figure 3).

### 3.7. Comparison of Swallowing Function before and after Treatment between Two Groups

There was no significant difference in the MDADI score between the two groups before treatment (*P* > 0.05). However, after intervention, the MDADI score increased significantly in both groups (*P* < 0.05) and was higher in the observation group compared with the control group (*P* < 0.05) (Table 4).

### 3.8. Comparison of Negative Emotion Scores between Two Groups before and after Treatment

The SDS and SAS scores were not significantly different between the two groups before treatment (*P* > 0.05). While after treatment, the two scores decreased significantly in both groups (*P* < 0.05) and were lower in the observation group compared with the control group (*P* < 0.05) (Figure 4).

### 3.9. Comparison of Life Quality Scores between Groups after Treatment

After treatment, patients in the observation group patients gained a markedly higher score on life quality than those in the control group in terms of physical status, psychological status, social relationships, life status, and level of independence (*P* < 0.05) (Table 5).

## 4. Discussion

Stroke is a common clinical cerebrovascular disease characterized by sudden attack of blood circulation disorders in the brain. Cerebral vascular blockage, rupture, and ischemia caused by internal carotid artery, vertebral artery atherosclerosis, arterial intimal hyperplasia, hypertrophy, and carotid artery trauma are the pathological basis of stroke [20]. Stroke is characterized by fast onset, high disability, and fatality rate. However, data show that as long as rehabilitation measures are taken in time when the motor cortex of a stroke patient is injured, the recovery of the patient's neurological function and activities of daily living can be accelerated [21]. Rehabilitation therapy can guide patients to actively practice their injured parts and functional activities, which in turn promotes the reconstruction of brain function, facilitating the recovery of muscles of the affected side, whereas single treatment still has shortcomings and needs to be combined with other treatments for better efficacy [22]. Acupuncture and moxibustion have the functions of refreshing the brain and resuscitating, invigorating the circulation of qi, strengthening joints, activating blood and removing blood stasis, and clearing channels and collaterals. Acupoint massage can promote local blood circulation, relieve limb spasm, and stimulate sensory nerve function recovery [23]. In the present study, we analyzed the effects of rehabilitation therapy combined with acupuncture on stroke patients.

RETRACTED

First, we compared the neurological deficits of patients between the two groups, and the results showed that the neurological recovery of the observation group was better than that of the control group. The efficacy evaluation results also showed that the observation group had a significantly higher ORR than the control group, suggesting that acupuncture combined with rehabilitation therapy could further alleviate neurological deficits. Then, plasma Cor and NPY levels were also compared before and after treatment. Elevated NPY levels can cause strong cerebral vasoconstriction, resulting in reduced local blood flow in the brain and aggravating the severity of the disease [24]. In addition, the neuroendocrine system will be activated to release a large amount of Cor when the patient's body is abnormal. The increase of Cor indicates the patient has a strong emergency response, which is likely to cause symptoms of cerebral hemorrhage [25]. In this study, it was observed that plasma levels of Cor and NPY in the observation group were lower than those in the control group after treatment, indicating that traditional Chinese acupuncture combined with rehabilitation therapy could effectively improve the neurological function of stroke patients, which was also consistent with the previous results. According to the theory of syndrome differentiation treatment, acupuncture and moxibustion stimulation of meridians has the effects of refreshing and resuscitating, reducing swelling and removing blood stasis, relaxing muscles and collaterals, antagonizing the generation of free radicals, alleviating brain edema, inhibiting the body's immune inflammatory response, and reducing the release of excitatory amino acids [26]. The abovementioned roles of acupuncture and moxibustion can also explain our findings. Previous studies have found that the effect of acupuncture is essential in the subacute stage of ischemic stroke, as it can effectively improve the clinical efficacy of patients and alleviate neurological deficits in patients [27], which is consistent with our observations.

RETRACTED

Subsequently, we compared the motor function, self-care ability, balance ability, and swallowing function between the two groups. The swallowing function was significantly improved in both groups after treatment, especially in the observation group. Cerebral infarction can lead to brain damage and nerve function damage, and blood flow to the affected area or nervous system damage will cause a series of complications such as limb dysfunction, cognitive dysfunction, and swallowing dysfunction, while acupuncture can stimulate specific acupoints to regulate qi and blood and warm the meridians, thereby more effectively relieving the patient's dysfunction [28]. Besides, life and economic pressure caused by the disease will also have a series of negative effects on the mood of stroke patients, while a good curative effect is beneficial to patients with negative emotions. Therefore, in this study, we also compared the negative emotion scores between the groups. The results revealed that the SDS and SAS scores decreased significantly in both groups after treatment and were lower in the observation group compared with the control group. This suggested that the combination of acupuncture and rehabilitation therapy was more conducive to the emotional relief of patients. Finally, we compared the life quality between the two groups after treatment, and the results identified a better quality of life in the observation group. The reason may be that better curative effect contributed to better relief of negative mood, which in turn improved the treatment compliance of patients, thus creating a virtuous circle and contributing to improved quality of life of patients. Few studies have combined acupuncture and rehabilitation therapy or focused on a more comprehensive neurological evaluation on stroke patients. This study is the first to find that combining acupuncture and rehabilitation therapy could effectively improve the nerve function of stroke patients and alleviate their negative emotions.

## 5. Conclusion

In summary, acupuncture and moxibustion of traditional Chinese medicine combined with rehabilitation therapy have outstanding effects in the treatment of stroke and can effectually improve the neurological function, prognosis, and life quality of patients, which is worthy of clinical promotion. However, this study also has certain shortcomings. First, due to the small sample size, the research results need to be further verified with a large sample size. In the future, multicenter and large-sample research will be carried out to obtain more accurate research results. Second, this study failed to compare the efficacy of acupuncture at different acupoints. Therefore, the efficacy of acupuncture treatment, as well as the curative effect of acupuncture combined with different targeted rehabilitation treatment modes, needs to be further explored.

RETRACTED

## Figures and Tables

**Figure 1:** Comparison of plasma Cor and NPY levels between two groups before and after treatment. (a) Comparison of plasma Cor levels between two groups before and after treatment. (b) Comparison of NPY levels between two groups before and after treatment. ^∗^ indicates *P* < 0.05.

**Figure 2:** Comparison of motor function and self-care ability between two groups before and after treatment. (a) Comparison of motor function between two groups before and after treatment. (b) Comparison of self-care ability between two groups before and after treatment. ^∗^ indicates *P* < 0.05.

**Figure 3:** Comparison of BBS scores between two groups before and after treatment. ^∗^ indicates *P* < 0.05.

**Figure 4:** Comparison of negative emotion scores between two groups before and after treatment. (a) Comparison of SDS scores between two groups before and after treatment. (b) Comparison of SAS scores between two groups before and after treatment. ^∗^ indicates *P* < 0.05.

**Table 1:** General information table (*n* (%)).

ITEM	Observation group (*n* = 52)	Control group (*n* = 48)	*t*/*X*^2^	*P*
Gender			0.021	0.884
Male	30 (57.69)	27 (56.25)		
Female	22 (42.31)	21 (43.75)		
Age (years)			0.087	0.768
≤65	21 (40.38)	18 (37.50)		
>65	31 (59.62)	30 (62.50)		
BMI (kg/m^2^)			0.001	0.987
≤23	25 (48.08)	23 (47.92)		
>23	27 (51.92)	25 (52.08)		
Smoking history			0.013	0.909
Yes	20 (38.46)	19 (39.58)		
No	32 (61.54)	29 (60.42)		
Diabetes			0.001	0.974
Yes	28 (53.85)	26 (54.17)		
No	24 (46.15)	22 (45.83)		
Hypertension			0.043	0.835
Yes	26 (50.00)	25 (52.08)		
No	26 (50.00)	23 (47.92)		
Stroke type			0.005	0.946
Cerebral infarction	35 (67.31)	32 (66.67)		
Cerebral hemorrhage	17 (32.69)	16 (33.33)		

**Table 2:** Comparison of therapeutic effects between groups.

Therapeutic effect	Observation group (*n* = 52)	Control group (*n* = 48)	*X* ^2^	*P*
Markedly effective	30 (57.69)	22 (45.83)	—	—
Effective	20 (38.46)	16 (33.33)	—	—
Ineffective	2 (3.85)	10 (20.83)	—	—
Overall response rate	50 (96.15)	38 (79.17)	6.821	0.009

**Table 3:** Comparison of neurological deficit scores before and after treatment between groups.

When	Observation group (*n* = 52)	Control group (*n* = 48)	*t*	*P*
Before treatment	22.16 ± 2.7	22.44 ± 2.95	0.496	0.621
After treatment	11.24 ± 1.12	17.19 ± 1.23	25.32	<0.001

**Table 4:** Comparison of swallowing function between groups before and after treatment.

When	Observation group (*n* = 52)	Control group (*n* = 48)	*t*	*P*
Before treatment	51.67 ± 2.6	51.91 ± 2.25	0.494	0.623
After treatment	81.02 ± 2.2	70.91 ± 2.27	22.61	<0.001

RETRACTED

**Table 5:** Comparison of life quality scores of between two groups after treatment.

Items	Observation group (*n* = 52)	Control group (*n* = 48)	*t*	*P*
Physiological status	49.51 ± 2.19	42.46 ± 2.29	6.807	<0.001
Psychological status	71.01 ± 2.49	60.03 ± 2.12	23.65	<0.001
Social relationships	43.06 ± 1.93	35.32 ± 1.94	19.99	<0.001
Life status	78.71 ± 2.51	72.12 ± 2.1	14.18	<0.001
Level of independence	59.91 ± 2.32	53.04 ± 2.16	15.29	<0.001

## Data Availability

The simulation experiment data used to support the findings of this study are available from the corresponding author upon request.
